# Rosiglitazone Suppresses the Growth and Invasiveness of SGC-7901 Gastric Cancer Cells and Angiogenesis In Vitro via PPAR*γ* Dependent and Independent Mechanisms

This article has been retracted.

**DOI:** 10.1155/2008/649808

**Published:** 2008-09-15

**Authors:** Qing He, Ruiping Pang, Xin Song, Jie Chen, Huixin Chen, Baili Chen, Pinjin Hu, Minhu Chen

**Affiliations:** ^1^Department of Gastroenterology, The First Affiliated Hospital, Sun Yat-Sen University, Guangzhou 510080, China; ^2^Department of Gastroenterology, Gastroenterology Institute, The Sixth Affiliated Hospital, Sun Yat-Sen University, Guangzhou 510080, China; ^3^Department of Physiology, Zhongshan School of Medicine, Sun Yat-Sen University, Guangzhou 510080, China

## Abstract

Although thiazolidinediones (TZDs) were found to be ligands for peroxisome proliferators-activated receptor*γ* (PPAR*γ*), the mechanism by which TZDs exert their anticancer effect remains unclear. Furthermore, the effect of TZDs on metastatic and angiogenesis potential of cancer cells is unknown. Our results in this paper show that rosiglitazone inhibited SGC-7901 gastric cancer cells growth, caused G1 cell cycle arrest and induced apoptosis in a dose-dependent manner. The effects of rosiglitazone on SGC-7901 cancer cells were completely reversed by treatment with PPAR*γ* antagonist GW9662. Rosiglitazone inhibited SGC-7901 cell migration, invasiveness, and the expression of MMP-2 in dose-dependent manner via PPAR*γ*-independent manner. Rosiglitazone reduced the VEGF induced angiogenesis of HUVEC in dose-dependent manner through PPAR*γ*-dependent pathway. Moreover, rosiglitazone did not affect the expression of VEGF by SGC-7901 cells. Our results demonstrated that by PPAR*γ* ligand, rosiglitazone inhibited growth and invasiveness of SGC-7901 gastric cancer cells and angiogenesis in vitro via PPAR*γ*-dependent or -independent pathway.

## 1. INTRODUCTION

Peroxisome proliferator-activated receptor gamma (PPAR*γ*) is a member of the ligand-inducible nuclear receptor superfamily. After activation, PPAR*γ* associates with the 9-cis retinoic acid receptor (RXR) to form functional heterodimers, which binds to the PPAR response element of the target genes and regulates the expression of these genes. Previous documents have shown that the PPAR*γ*/RXR signal pathway plays critical role in a variety of biological processes, including adipogenesis, glucose metabolism, inflammation as well as inhibition of normal and tumor cells growth [1].

Thiazolidinediones (TZDs) are synthetic agonists for PPAR*γ*. These PPAR*γ* ligands were clinically used as antidiabetic drugs which could attenuate the insulin resistance associated with obesity, hypertension, and impaired glucose tolerance in humans [2]. Recent studies have suggested that PPAR*γ* is a potential molecular target for anticancer drug development, due to the increased expression of PPAR in several cancer cells. It has been reported that TZDs could inhibit growth and induce apoptosis in a variety of cancer cell lines. More importantly, TZDs exhibited antitumor activities in vivo in the prevention of prostate, liver, and pituitary cancers. Although increasing evidence showed that TZDs are potential anticancer agents [3], the mechanisms underlying the antitumor effects are not well understood. TZDs were initially thought to inhibit the cancer cells proliferation through regulation of expression of PPAR*γ*-mediated target genes. However, recent evidence revealed that the antitumor effects of TZDs exist via PPAR*γ*-independent mechanisms in various types of cancers [4–6].

We previously found the expression of PPAR*γ* decreased in primary and metastatic gastric carcinoma, compared with normal gastric tissues [7]. Recent studies in gastric cancer cells demonstrated that TZDs treatment resulted in significant growth arrest both in cultured cell and in nude mice models [8–12]; however, the effects of PPAR*γ* ligands on invasiveness and angiogenesis of gastric cancer are still unclear. Therefore, this work was undertaken to investigate the effects of PPAR*γ* agonists, such as rosiglitazone, on cell growth and the invasiveness in human cell line SGC-7901, as well as on angiogenesis in vitro. 

## 2. METHODS

### 2.1. Cell culture

Human gastric cancer cell line, SGC-7901, was obtained from the Type Culture Collection of Chinese Academy of Sciences (Shanghai, China). Human umbilical vein endothelial cells (HUVECs) were purchased from the Keygen Technology Company (Najing, China). SGC7901 cells and HUVECs were cultured in RPMI-1640 medium (GIBCO, Carlsbad, Calif, USA) containing 10% fetal bovine serum (FBS) and 1% antibiotics (100 U/mL penicillin G, 100 *μ*g/mL streptomycin sulfate, Sigma-Aldrich, Mo, USA).

### 2.2. RT-PCR

Total RNA was isolated using TRIzol Reagent (Invitrogen, Carlsbad, Calif, USA) according to the manufacturer's instructions. Reverse transcription reaction was performed with random hexamer primers and a SuperScript Reverse transcriptase kit (Invitrogen, Carlsbad, Calif, USA). The sequences of specific primers were as follows: PPAR*γ* mRNA, forward, 5′-TCT CTC CGT AAT GGA AGA CC-3′, and reverse, 5′-GCA TTA TGA GAC ATC CCC AC-3′. MMP-2 mRNA, forward, 5′-GGC CCT GTC ACT CCT GAG AT-3′, and reverse, 5′-GGC ATC CAG GTT ATC GGG GA-3′. VEGF mRNA, forward, 5′-GAC AAg AAA ATC CCT GTG GGC-3′, and reverse 5′-AAC GCG AGT CTG TGT TTT TGC-3′. *β*-actin mRNA, forward, 5′-CTT CTA CAA TGA GCT GCG TA-3′, and reverse, 5′-TCA TGA GGT AGT CAG TCA GG-3′. PCR conditions were 94°C, 30 seconds, 55–57°C (depending on the primer set), 30 seconds, and 72°C, 1 minute with 35 cycles using Taq PCR MasterMix (Tianwei, Beijing, China). The resultant PCR products were 474 bp (PPAR*γ*), 243 bp (*β*-actin), 474 bp (MMP-2), and 169 bp (VEGF). PCR products were electrophoresed on a 1.2% agarose gel and visualized by ethidium bromide staining.

### 2.3. Quantitative real-time RT-PCR analysis

The PCR reactions were performed in a Brilliant SYBR Green QPCR master mix (Stratagene, Calif, USA) according to the manufacturer's instructions. The sequences of specific primers were the same as for RT-PCR. After 10 minutes at 95°C to denature the cDNA, the cycling conditions were 95°C, 1 minute, 55–57°C (depending on the primer set), 30 seconds, and 72°C, 1 minute with 40 cycles. The LightCycler software constructed the calibration curve by plotting the crossing point (Cp), and the numbers of copies in unknown samples were calculated by comparison of their Cps with the calibration curve. To correct differences in both RNA quality and quantity between samples, the data were formalized to those for *β*-actin.

### 2.4. Western blotting

The cells proteins were extracted according to NE-PER Nuclear and Cytoplasmic Extraction Reagents kit (Pierce, Rockford, Ill, USA). Protein concentration of each sample was assayed using BCA Protein Assay Reagent according to manufacturer's instructions (Pierce Biotechnology, Rockford, Ill, USA). Twenty micrograms of proteins of different groups were separated in 10% SDS-PAGE, and transferred onto PVDF membrane (Invitrogen, Carlsbad, Calif, USA). Five percent of milk (blocking solution) was loaded over the membrane and incubated for 1 hour at room temperature with agitation. The membranes were then incubated with the mouse antihuman PPAR*γ* antibody at a dilution of 1:200 (Santa Cruz, Calif, USA), the mouse antihuman MMP-2 antibody (1:400, Neomarker, Calif, USA), the rabbit antihuman VEGF antibody (1:200, Zymed, Calif, USA), and the mouse antihuman *β*-actin (1:200, Xiaxin, China) overnight at 4°C with agitation. After being washed with 0.1% Tween 20 in Tris-saline, three times, the membranes were incubated with biotin-labeled antirabbit or mouse IgG for 1 hour at room temperature with agitation. Reactive protein was detected using ECL chemiluminescence system (Pierce, Rockford, Ill, USA).

### 2.5. ELISA of secreted VEGF

The effect of RGZ on VEGF release in tumor cells was measured by ELISA. Cells grown in 90 mm plates were exposed to various concentrations of RGZ (1–20 *μ*M) or vehicle with or without GW9662 (2.5 *μ*M, pretreated 1 hour) for 24 hours. VEGF concentration in the supernatant was measured using a VEGF ELISA kit (R & D systems, Minneapolis, Minn, USA).

### 2.6. Cell viability

The viability of the cells was assessed by MTT assay. Briefly, cells grown in 96-wells were exposed to various concentrations of RGZ with or without GW9662 (2.5 *μ*M, pretreated 1 hour), for 24, 48, or 72 hours. Then, 20 *μ*L of MTT (5 mg/mL) was added to each well, and cells were incubated continuously at 37°C for 4 hours. After removal of medium, the crystals were dissolved in DMSO, and absorbance was assessed at 570 nm with a microplate reader.

### 2.7. Cell cycle and apoptosis analysis

Cells treated with RGZ (1–20 *μ*M) or vehicle with or without GW9662 (2.5 *μ*M, pretreated 1 hour) for 48 hours were collected and fixed in cold 70% ethanol. Then, the samples were treated with RNase, stained with 50 mg/mL propidium iodide (PI), and analysed by EPICS Elite flow cytometer (Coulter Electronics, Fla, USA).

### 2.8. Invasion assay

The ability of cells to invade through a Matrigel-coated filter was measured in transwell chambers (Corning, NY, USA). Polyvinylpyrrolidone-free polycarbonate filters (pore size 8 *μ*m) were coated with basement membrane Matrigel (50 *μ*L/filter) (BD, Bedford, Ohio, USA). The membrane was washed in PBS to remove excess ligand, and the lower chamber was filled with 0.6 mL of RPMI-1640 medium containing 10% fetal bovine serum (FBS). Cells were serum-starved overnight (0.5% FBS), harvested with trypsin/EDTA, and washed twice with serum-free RPMI-1640 medium. Cells were resuspended in migration medium (RPMI-1640 medium with 0.5% FBS), and 0.1 mL migration medium containing 1 × 10^5^ cells was added to the upper chamber. After incubation with RGC (1–20 *μ*M) with or without GW9662 (2.5 *μ*M, pretreated 1 hour) at 37°C for 24 hours, the cells on the upper surface of the membrane were removed using a cotton swab. The migrant cells attached to the lower surface were fixed in 10% formalin at room temperature for 30 minutes and stained with hematoxylin. The numbers of migrated cells were counted under a microscope.

### 2.9. Scratch wound-healing motility assays

Gastric cancer cells were seeded on 60 mm plates and allowed to grow to confluence. Confluent monolayers were scratched with a pipette tip and maintained under RGZ (1–20 *μ*M) with or without GW9662 (2.5 *μ*M, pretreated 1 hour) for 24 hours. Plates were washed once with fresh medium to remove nonadherent cells and then photographed. The cell migration was evaluated by counting cells that migrated from the wound edge.

### 2.10. In vitro Angiogenesis assay

The angiogenesis assays were performed as per the manufacturer's instructions, that is, transfer 50 *μ*L of ECMatrixTM solution to each well of a precooled 96-well tissue culture plate on ice. Incubate at 37°C for 1 hour to allow the matrix solution to solidify. Harvest human umbilical vein endothelial cells (HUVECs) resuspend and Seed 5 × 10^3^ cells per well onto the surface of the polymerized ECMatrixTM. Incubate with RGC (1–20 *μ*M) with or without GW9662 (2.5 *μ*M, pretreated 1 hour) at 37°C for 12 hours. Inspect tube formation under an inverted light microscope at 100 X magnification.

### 2.11. Zymography

Cells were cultured for 24 hours in serum-free medium, washed twice, and finally treated with RGZ (1–20 *μ*M) with or without GW9662 (2.5 *μ*M, pretreated 1 hour) for a further 48 hours. The supernatants were collected and concentrated, using centrifugal filter devices (Millipore Corp., Bedford, Mass, USA) and the protein content was determined using BCA Protein Assay Reagent. Equal amounts of protein (20 *μ*g) were mixed with SDS sample buffer without reducing agents and incubated for 40 minutes at 37°C. For gelatinolytic activity, the assay samples were separated on polyacrylamide gels containing 1mg/mL gelatin. After electrophoresis, the gels were stained for 1 hour in a 45% methanol/10% acetic acid mixture containing coomassie brilliant blue G250 and destained. Zymograms were photographed after 10 hours of incubation at 37°C.

### 2.12. Statistical analysis

Data are expressed as mean ± standard deviation (SD) of three independent experiments, each done in triplicate. Differences between control and experiment groups were analyzed using the *t*-test. *P* < .05 was considered statistically significant.

## 3. RESULTS

### 3.1. RGZ inhibited proliferation and induced apoptosis in SGC-7901 cells through PPAR*γ*-dependent mechanism

In SGC-7901 cells, the expression of PPAR*γ* was observed by RT-PCR and western blot (not shown).

RGZ (0.1–100 *μ*M) treatment for 24, 48, and 72 hours inhibited cells growth in a dose- and time-dependent manners in SGC-7901 gastric cancer cell line as determined by MTT assay. Pretreatment with the highly selective PPAR*γ* antagonist GW9662 (2.5 *μ*M) reversed the effect of RGZ on cell viability (see Figure 1(a)).

To explore whether the growth inhibition of RGZ in SGC-7901 cells was caused by apoptosis, we analyzed the sub-G1 population of the cells after treatment with RGZ (1–20 *μ*M) for 48 hours. RGZ induced apoptosis in a dose-dependent manner, which was also reversed completely by 2.5 *μ*M GW9662 treatment (see Figure 1(b)).

Furthermore, to determine whether the inhibitory effect of RGZ on cell viability is associated with the arrest of the cell cycle, we analyzed the cell cycle progression after treatment with RGZ (1–20 *μ*M) for 48 hours. RGZ treatment increased the number of cells in the G1-G0 and decreased the number of cells in the S phases in dose-dependent manner. The effects of RGZ on cell cycle of SGC-7901 cells were also reversed by 2.5 *μ*M GW9662 (see Figure 1(c)).

### 3.2. RGZ inhibited SGC-7901 cells migration and invasiveness through PPAR*γ*-independent mechanism

After treatment with RGZ (1–20 *μ*M) for 48 hours, the number of cells migrated to the scratched area was 60 ± 3.1 cells/mm^2^, 58 ± 2.7 cells/mm^2^, 49 ± 2.8 cells/mm^2^, 27 ± 2.9 cells/mm^2^, and 20 ± 1.9 cells/mm^2^, respectively, which were significantly lower than those in control group (84 ± 3.4 cells/mm^2^). GW9662 treatment had no effects on the cells migration with inhibition induced by RGZ. The number of the cells migrated to the scratched area treated with GW9662 and RGZ (1–20 *μ*M) for 48 hours was 61 ± 1.8 cells/mm^2^, 53 ± 3 cells/mm^2^, 47 ± 2.5 cells/mm^2^, 29 ± 2.8 cells/mm^2^, 18 ± 3.2 cells/mm^2^, respectively, which were not different from those in the groups treated with RGZ alone (see Figure 2(a)).

The effect of RGZ on the cells invasion through reconstituted basement membranes was analyzed using Matrigel-coated invasion chambers. After treatment with RGZ (1–20 *μ*M) for 48 hours, the cells attached to the lower surface of the filters were 256 ± 9 cells/mm^2^, 248 ± 7 cells/mm^2^, 219 ± 12 cells/mm^2^, 174 ± 11 cells/mm^2^, and 154 ± 10 cells/mm^2^, respectively, which were significantly lower than those in control group (279 ± 9 cells/mm^2^). After cotreatment of the cells with GW9662 and RGZ, the cells attached to the lower surface were 251 ± 29 cells/mm^2^, 238 ± 12 cells/mm^2^, 220 ± 7 cells/mm^2^, 166 ± 16 cells/mm^2^, and 148 ± 12 cells/mm^2^, respectively, which were not different from those in the groups treated with RGZ alone (see Figure 2(b)).

Metalloproteases (MMPs) have been demonstrated to play a significant role in tumor cell invasion [13]. In this study, our results showed that RGZ inhibited the mRNA and protein expression levels of MMP-2 in a dose-dependent manner (see Figures 3(a), 3(c), and Tables 1, 2). Moreover, the gel zymography results demonstrated that the activity of MMP-2 decreased after RGZ (1–20 *μ*M) treatment for 48 hours in dose-dependent manner (see Figure 4(a)). The inhibitory effects of RGZ on MMP-2 were not affected by GW9662 treatment (see Figures 3(b), 3(c), and 4(b)).

### 3.3. Effects of RGZ on angiogenesis in vitro

Matrigel-plated HUVECs elongated and migrated in the presence of VEGF and formed tubular networks. RGZ markedly suppressed the formation of the tube-like structures of HUVEC cells in a dose-dependent manner (see Figure 5(a)), which was completely antagonized by GW9662 (see Figure 5(b)). These results suggested that rosiglitazone exhibits antiangiogenic activity via PPAR*γ*-dependent mechanism.

To further determine whether the effect of RGZ on angiogenesis is due to the down regulation of the tumor-secreted growth factors, we measured the expression levels of VEGF in SGC-7901 cell cultured medium, after treatment with various concentrations of RGZ. Our results demonstrated that RGZ (1–20 *μ*M) did not change the expression of mRNA and protein of VEGF in SGC-7901 cells (see Figures 3(a), 3(c), and Table 1), but also the results were confirmed by ELISA (see Figure 6).

## 4. DISCUSSION

As a potential molecular target for anticancer drug development, PPAR*γ* and its ligands have been extensively studied in the past several years. Previous studies have shown that PPAR*γ* is expressed in several human gastric-cancer cell lines, including MKN-7, MKN-28, MKN-45, and AGS. TZDs could inhibit these cancer cell lines growths in vitro and in vivo [9, 12]. Also, the growth inhibitory effects of TZDs on MKN45 cells depend on the PPAR*γ* expression levels. The growth inhibition of TDZs was more significant in the higher PPAR*γ* expressing cells. Moreover, Lu et al. [10] found that PPAR*γ* (+/ − ) mice were more susceptible to MNU-induced gastric cancer than wild-type (+/+) mice, and troglitazone significantly reduced the incidence of gastric cancer in PPAR*γ* (+/+) mice but not in PPAR*γ* (+/ − ) mice. All these results indicated that TZDs inhibit the cancer cells growth via PPAR*γ*-dependent mechanism. Our results demonstrated that RGZ, the most potent and selective synthetic ligand of PPAR*γ*, inhibited SGC-7901 gastric cancer cells growth, caused G1 cell cycle arrest, and induced apoptosis in a dose-dependent manner. The effects of RGZ on SGC-7901 cancer cells were completely reversed by treatment with PPAR*γ* antagonist GW9662. These results indicated that RGZ suppressed the SGC-7901 cancer cells growth in a PPAR*γ*-dependent mechanism.

In this study, we found that the RGZ inhibited invasion, migration, and the secretion of MMP-2 of SGC-7901 cells. The inhibitory effects of RGZ on metastases and MMP-2 activity were not directly mediated by PPAR*γ* activation, since these effects were not reversed by GW9662 treatment. Our results were consistent with the previous works on human adrenocortical cancer cell line H295R [14], pancreatic cancer cells [15], and human myeloid leukemia cells [16], which showed that PPAR*γ* ligands act independently of PPAR*γ* activation in the invasion suppression and down-regulation of MMP-2 activity. Recent papers showed that PPAR*γ* regulated E-cadherin expression and inhibited growth and invasion of prostate cancer [17], and PPAR*γ* ligand troglitazone inhibited transforming growth factor-beta-mediated glioma cell migration and brain invasion [18]. But some studies have contrasting results that the PPAR*γ*, ciglitazone, induced cell invasion, through activation of Pro-MMP-2, activation via the generation of ROS, and the activation of ERK [19], and that PPAR*γ* antagonists induced vimentin cleavage and inhibited invasion in high-grade hepatocellular carcinoma [20]. Further studies are needed on the mechanism of PPAR*γ* in cancer and invasion.

Recent investigations suggested that PPAR*γ* ligands had inhibitory effects on tumor cell lines, but the effects appear not to be entirely elicited by the direct action on tumor cells. Inhibition of the neovascularization may be another target of TZDs to suppress the growth of cancers. PPAR*γ* is expressed in endothelial cells, and the PPAR*γ* ligands can inhibit the proliferation of these cells induced by growth factors, or cause their apoptosis in vitro [21–23]. It has been reported that PPAR*γ* ligands could inhibit choroidal, retinal, and corneal neovascularization when administered intraocularly [24–26]. In addition, systemic administration of rosiglitazone and troglitazone inhibits FGF2-induced angiogenesis; thereby inhibiting primary tumor growth and metastasis [27]. We observed that RGZ inhibited the angiogenesis of HUVECs in dose-dependent manner via PPAR*γ* pathway. The effects RGZ on the endothelium suggest that RGZ may regulate tumor growth by targeting non-cell-autonomous mechanisms.

Previous studies [5] showed that suppression of angiogenesis could result from a decrease in the local levels of stimulators (e.g., VEGF and FGF2) and/or an increase of endogenous inhibitors of angiogenesis (e.g., thrombospondin) produced by tumor cells. PPAR*γ* ligands suppressed VEGF production in colon carcinoma [28], human breast cancer [29], and human renal cell carcinoma cells [30]. However, contradictory results have also been reported in bladder and prostate cancer cells in which PPAR*γ* ligands increased VEGF production [31, 32]. Inconsistent with the above documents, our results showed that RGZ did not change the secretion of VEGF from SGC-7901.

Taken together, our results demonstrated that RGZ inhibited growth and invasiveness of SGC-7901 gastric cancer cells and angiogenesis in vitro via PPAR*γ*-dependent or -independent pathway. Further study is needed to elucidate the mechanisms by which RGZ exhibits different manner.

## Figures and Tables

**Figure 1:** (a) RGZ (0.1–100 *μ*M) treatment for 24, 48, and 72 hours inhibited cell growth in a dose- and time-dependent manners in SGC-7901 gastric cancer cell line, as determined by MTT assay, which was reversed completely by 2.5 *μ*M GW9662 pretreatment for 1 hour. Cell viability was expressed as the percentage of cells under control conditions (0 *μ*M of RGZ or GW9662). (b) RGZ induced apoptosis in a dose-dependent manner, which was also reversed completely by 2.5 *μ*M GW9662 pretreatment for 1 hour. (c) RGZ treatment increased the number of cells in the G1-G0 and decreased the number of cells in the S phases in dose-dependent manner, which was reversed completely by 2.5 *μ*M GW9662 pretreatment for 1 hour. Values are the means ± SD of three representative experiments.*Statistical significance (*P* < .05 or higher degree of significance) versus vehicle-treated controls.

**Figure 2:** (a) Effect of RGZ on the migration and (b) invasion of SGC-7901 gastric cancer cells, which was reversed completely by 2.5 *μ*M GW9662 pretreatment for 1 hour. Values are the means ± SD of three representative experiments.*Statistical significance (*P* < .05 or higher degree of significance) versus vehicle-treated controls.

**Figure 3:** (a) RGZ (1–20 *μ*M) inhibited the mRNA and (c) protein expression levels of MMP-2 in a dose-dependent manner, which were not affected by 2.5 *μ*M GW9662 pretreatment for 1 hour (b), (c). RGZ (1–20 *μ*M) did not change the expression of VEGF in SGC-7901 cells (a), (c).

**Figure 4:** (a)The activity of MMP-2 was decreased after RGZ (1–20 *μ*M) treatment for 48 hours in dose-dependent manner. (b) The inhibitory effects of RGZ on MMP-2 were not affected by 2.5 *μ*M GW9662 pretreatment for 1 hour.

**Figure 5:** (a) RGZ markedly suppressed the formation of the tube-like structures of HUVEC cells in a dose-dependent manner, (b) which was completely antagonized by 2.5 *μ*M GW9662 pretreatment for 1 hour.

**Figure 6:** RGZ had no effect on the secretion of VEGF of SGC-7901 cell.

**Table 1:** Expression of MMP-2 and VEGF after RZD treatment in SGC-7901 gastric cancers by real-time PCR.

Rosiglitazone (*μ*mol/L)	PPAR*γ*	MMP-2	VEGF
0	0.132127 ± 0.045513	0.008912 ± 0.000133	0.61132 ± 0.078921
1	0.121878 ± 0.034219	0.006003 ± 0.000331*	0.620255 ± 0.054671
3	0.130134 ± 0.0521137	0.005486 ± 0.000541*	0.60728 ± 0.036799
5	0.137778 ± 0.046222	0.005048 ± 0.000346*	0.599438 ± 0.076541
10	0.141171 ± 0.038741	0.001924 ± 0.000189*	0.624165 ± 0.038966
20	0.143889 ± 0.061237	0.001298 ± 0.000267*	0.604246 ± 0.065679

*Statistical significance (*P* < .05 or higher degree of significance) versus vehicle-treated controls.

**Table 2:** Expression of MMP-2 and VEGF after RZD and GW9662 cotreatment in SGC-7901 by real-time PCR.

Rosiglitazone (*μ*mol/L)	PPAR*γ*	MMP-2
0	0.14161 ± 0.055389	0.00975 ± 0.000533
1	0.137738 ± 0.030102	0.008974 ± 0.000113*
3	0.134614 ± 0.029881	0.006003 ± 0.000401*
5	0.141156 ± 0.564569	0.00564 ± 0.000246*
10	0.135666 ± 0.034887	0.002182 ± 0.000364*
20	0.129278 ± 0.019262	0.001712 ± 0.000178*

*Statistical significance (*P* < .05 or higher degree of significance) versus vehicle-treated controls.
